The article "China's Economic Forecast Based on Machine Learning and Quantitative Easing" was published in 2022. Journal: Comput Intell Neurosci.

# China's Economic Forecast Based on Machine Learning and Quantitative Easing

**DOI:** 10.1155/2022/2404174

**Published:** 2022-03-26

**Authors:** Chang Qiu

**Affiliations:** School of Statistics and Management, Shanghai University of Finance and Economics, Shanghai 200433, China

## Abstract

In this paper, six variables, including export value, real exchange rate, Chinese GDP, and US IPI, and their seasonal variables, are used as determinants to model and forecast China's export value to the US using three methods: BP neural network, ARIMA, and AR-GARCH. Error indicators were chosen to compare the simulated and predicted results of the three models with the real values. It is found that the results of all three models are satisfactory, although there are some differences in their simulation and forecasting capabilities, but the ARIMA model has a clear advantage. This paper analyses the reasons for these results and proposes suggestions for improving China's exports in the context of the models.

## 1. Introduction

Export trade is one of the driving forces behind China's rapid economic growth, and the United States, as China's top export trading partner, has a huge impact on China's economic development. However, recently, due to the global economic crisis and the appreciation of the RMB against the USD, China's export growth has started to slow down and even become negative. Therefore, modelling China's exports to the US and quantifying the factors that influence them is extremely important in order to predict and take measures to increase China's export value [1].

Quantitative easing has been in place for many years, but the theoretical basis for this so-called unconventional policy has not yet been agreed upon by academics, and there is still much disagreement. In addition to the “liquidity trap theory,” many believe that the “non-neutral money theory,” “financial accelerator theory,” and the “great depression theory” proposed by Bernanke and others are the theoretical foundations of this policy. The “great depression theory” proposed by Bernanke and others also forms the theoretical basis for quantitative easing [2]. As a result of the implementation of quantitative easing, his theories are considered to be the veritable foundation of quantitative easing. However, the relationship between MMT and quantitative easing has been highlighted by the academic hype about modern monetary theory (MMT), the great recession and the implementation of unlimited quantitative easing, i.e., the former is the theoretical basis of the latter and the latter is the concrete practice of the former [3]. At present, academics have basically reached a consensus on whether MMT belongs to the theoretical basis of quantitative easing policy, but there is a greater controversy over the understanding of quantitative easing policy itself and its theoretical basis. Some domestic scholars who hold opposing views believe that MMT has major theoretical flaws and its basic proposition is a serious departure from reality, and thus a fallacy. The quantitative easing policy based on this theory also has major flaws, as it is essentially a kind of monetisation of fiscal deficits, in which fiscal expenditure is regarded as money creation and fiscal revenue is regarded as money recovery [4]. This is essentially an act of “robbing the poor to give to the rich” and “pulling the wool over the world's eyes.” Some mainstream economists abroad have also taken a negative view of MMT, arguing that it is both detrimental to the development of economic theory and harmful to real economic policy. Some scholars, however, are enthusiastic about the theoretical claims of MMT, arguing that it is a disruptive theoretical innovation, a fundamental rejection of mainstream macrofinance and fiscal theory, and even a solution to a major problem in the field of political economy.

The article "China's Economic Forecast Based on Machine Learning and Quantitative Easing" was published in 2022. Journal: Comput Intell Neurosci.

The author believes that whether the theoretical basis of quantitative easing policy is scientific or not must not only be tested by practice but also evaluated from the perspective of Marxist political economy. Therefore, based on the effectiveness of quantitative easing policy in the US, this paper systematically analyses the relationship between the operation process of quantitative easing policy and its theoretical basis, discusses the trend of normalisation of quantitative easing policy and its limitations from the perspective of Marxist political economy, makes necessary arguments on the internal link between quantitative easing policy and MMT, and points out the importance of conducting this study to China's understanding of quantitative easing policy and the formulation of policies to cope with the current round of the great recession. The study is also useful for China to understand quantitative easing and formulate policies to cope with the current round of the great recession [5].

## 2. Related Work

In the existing export trade forecasting literature, the main quantitative forecasting methods are ARIMA models, AR-GARCH models, neural network modelling methods, and some extensions based on them. Of these, the ARIMA and AR-GARCH models are upgrades of traditional time series models (exponential smoothing, moving average, etc.), and these linear forecasting methods have the advantage of being simple, intuitive, and highly explanatory. There is also a small body of literature on export trade forecasting using cointegration models, support vector machine models, and grey system methods. In terms of variable selection, the usual empirical variables are often used: export value variables, real exchange rate variables, GDP variables of importing and exporting countries, and their lagged variables. In addition, since macrovariables tend to be highly seasonally cyclical, they are generally seasonally adjusted in the literature [6].

The article "China's Economic Forecast Based on Machine Learning and Quantitative Easing" was published in 2022. Journal: Comput Intell Neurosci.

The empirical evidence is as follows: Yildirim and Ivrendi [7] extend the univariate ARMA model to multiple variables and test the model's effectiveness with forecasts of export effects for Sweden. A univariate ARIMA model based on a Bayesian search algorithm is presented in [7], which is empirically shown to be less effective in predicting seasonal models than nonseasonal models. In [8], a neural network model was used to forecast the export of DOC in Scotland, and methods such as increasing the sample size and improving the parameters were proposed to improve the accuracy of the model.

The ARIMA model was developed using the monthly export data of China from 2015 to 2021, with lagged export data as the determinant variable, trend differencing and seasonal differencing, and was used to forecast China's exports in 2023. [9] An AR-GARCH model was developed to simulate China's exports to the US using empirical variables as determinants and excluding seasonal effects, and a dynamic conditional correlation coefficient (DCC) model was used to analyse the impact of RMB appreciation on exports. Fofack et al. [10] analyse the application of cointegration techniques and error correction models based on them in forecasting, propose a nonlinear error correction forecasting model based on neuronal networks, combining the characteristics of neuronal networks, and forecasts the general situation of China's export trade in 2023. [11] An empirical analysis of Hunan Province's exports was conducted and the model was found to be effective in forecasting regional export trade.

In a comparative analysis of these methods, Cole et al. [12] used a neural network model, exponential smoothing, and ARIMA to forecast Thai rice exports and evaluated the effectiveness of the three methods using various indicators. Woo and Zhang [13] compared the advantages and disadvantages of the ARCH family model and the BP neural network model in predicting maize and stock prices, and both concluded that the nonlinear system modelling was slightly better than the linear model.

## 3. Basic Principles of the Three Models

### 3.1. Basic Principles of BP Neural Networks

A BP network is a multilayer feed-forward network with backpropagation of errors and is the most representative and widely used type of an artificial neural network. To train a BP network, the same set of inputs and desired outputs are used as training “samples,” and the network is trained according to a certain algorithm, and once trained, the model can be used to solve similar problems. A BP network requires a training set and a test set to evaluate its training results. The former is used to train the network to achieve a specified error, and the latter is used to evaluate the performance of the trained network.

The article "China's Economic Forecast Based on Machine Learning and Quantitative Easing" was published in 2022. Journal: Comput Intell Neurosci.

### 3.2. Fundamentals of the ARIMA Model

The ARIMA model, also known as the differential autoregressive moving average model, is an extension of the ARMA (p, q) model. In ARIMA (m, *d*, n), AR is the ‘autoregressive,' *m* is the number of autoregressive terms; MA is the ‘sliding average,' *n* is the number of sliding average terms, and *d* is the number of differences (orders) made to make it a smooth series. After *d* differences, the ARIMA (p, *d*, q) model can be expressed as an ARMA model with the following expression:

(1) $$\begin{array}{c} r_{t}=c+\sum_{i=1}^{m}\phi_{i}r_{t-i}+\sum_{j=1}^{n}a_{j}y_{t-j}+\varepsilon_{t}, \end{array}$$

where *r*_*t*−*i*_ is the *r*_*t*_ lagged i-order variable, *y*_*t*−*j*_ is the moving average term at lag *j*, and *ε*_*t*_ is the residual, which follows a standard normal distribution.

### 3.3. Fundamentals of the AR-GARCH Model

To describe and predict volatility clustering in economic time series, an autoregressive conditional heteroskedasticity model (i.e. ARCH model) is used. Since the ARCH model is a short memory process, in order to better characterise certain financial market phenomena with long memory processes, the authors of [14] generalises the ARCH model and adds lags to the residual term conditional variance to derive a generalised autoregressive conditional heteroskedasticity model (GARCH model). AR-GARCH is the addition of an autoregressive term to the mean expression of the GARCH model, which can be expressed as

(2) $$\begin{array}{c} r_{t}=c+\sum_{i=1}^{m}\phi_{i}r_{ti}+\varepsilon_{t},\\ \sigma_{t}^{2}=\omega +\sum_{i=1}^{p}\alpha_{i}\sigma_{t-i}^{2}+\sum_{j=1}^{q}\beta_{j}\sigma_{t-j}^{2}, \end{array}$$

where *r*_*t*_ is the series of returns, *σ*_*t*_^2^ is the series of variances, and *ε*_*t*_ is the residuals, and it follows a standard normal distribution.

## 4. Application of the Model and Empirical Analysis

### 4.1. Selection of General Variables

The most commonly used explanatory variables for the export function in the literature on exchange rate exports are: real exports with a lag; the real exchange rate; the GDP of the exporting country, which is a measure of the exporting country's export capacity; and the GDP (gross domestic product) of the importing country or other proxy variables (such as the industrial production index IPI), which are a measure of the importing country's import capacity.

The article "China's Economic Forecast Based on Machine Learning and Quantitative Easing" was published in 2022. Journal: Comput Intell Neurosci.

The lagged real exports are usually selected with a one-period lag, and in this paper, we also select a one-period lagged variable for China's exports to the US.

The real exchange rate is calculated using the formula

(3) $$\begin{array}{c} \text{real exchange rate}=\frac{\text{nominal exchange rate }x\text{ foreign price}}{\text{local currency commodity price}}. \end{array}$$

Foreign prices and local currency commodity prices are expressed in terms of the consumer price index (CPI) for both countries. The GDP data for China and the US are actually only available on a quarterly basis, and the sample for this paper is based on a monthly interval (if the interval is annual, then the data can be collected over a shorter period of time and the sample size is smaller), so I have tried to replace the data with monthly IPI data. As there has been no IPI data for China since 2006, this paper can only average the quarterly GDP data for China over three months to obtain monthly GDP data, while the IPI data are used to replace the US GDP data.

### 4.2. Selection of Seasonal Variables

As macrodata tends to be highly seasonal, the graphical analysis of the sample series shows that there is strong seasonality in the value of exports to the US and China's GDP. Exports, for example (Figure 1), have a strong annual cycle of their own, with the value of exports generally increasing, but suddenly decreasing in January and February each year, and then increasing again. China's GDP is also seasonal, and this is more pronounced in China (Figure 1). This is strongly related to the Chinese New Year holiday. So, in the forecasting model, we add seasonal lags to these two variables, i.e., the value of exports in the same period last year and the value of Chinese GDP in the same period last year, as determinants. This allows the model to capture the impact of seasonality on exports to the US and China's GDP.

In forecasting models, the dependent variable is usually replaced by a number of periods lagged, as data for the current independent variable is often not yet available for the forecast period. Therefore, the values of all decision variables in this model are brought into the model with a one-period lag. The six input variables of the input layer of this neural network prediction model are summarised in Figure 2.

### 4.3. Data Sources and Data Processing

Monthly data from 2015 to 2021 are used as sample data to model China's exports to the US. The nominal exchange rate of the RMB to the USD is obtained from the website of the State Administration of Foreign Exchange (SAFE); data on China's export trade to the US and China's Consumer Price Index (CPI) are obtained from the RESET database, while data on the US CPI and the Industrial Price Index (IPI) are obtained from the US Bureau of Labor Statistics and the Federal Reserve website.

The article "China's Economic Forecast Based on Machine Learning and Quantitative Easing" was published in 2022. Journal: Comput Intell Neurosci.

To calculate the real exchange rate, the ratio of the CPI indices for China and the US over the sample period is required. Since the US CPI is a chain index and the Chinese CPI (used in this paper) is a year-on-year index, we first convert the CPI data for each country into a CPI-based index based on the CPI index of January 2005.

### 4.4. Development of a BP Neural Network Model for Export Forecasting

There are three main stages in building a neural network model and completing training and learning: the configuration stage, the training stage, and the output stage.

We have already identified the factors that influence export value, with six main variables to be considered (Figure 2), which we will use as input nodes to the BP model. The input nodes are normalised to the indicator data by the following formula:

(4) $$\begin{array}{c} X^{\prime }=\frac{\left(x-x_{\min}\right)}{\left(x_{\max}-x_{\min}\right)}. \end{array}$$

The number of hidden layers and the number of nodes in the hidden layer are chosen as one layer. The number of nodes is directly related to the number of input and output units, which is determined by the formula $n1=\sqrt{n+m}+a$, where *m* is the number of input neurons equal to 6, *n* is the number of output neurons of 1, and *a* is a constant between 1 and 10. In this paper, after repeated debugging, the number of nodes in the hidden layer was determined to be 10.

Output node is the variable to be predicted, the value of China's exports to the US, which is also normalised here.

This stage completes the training of the network on the sample. For the input information, the neural network is propagated forward to the nodes in the implicit layer,and then transferred to the output node after a sigmoid-type activation function. The sigmoid function expression is *y*=1/(1+*e*^−*x*/*β*^) adaptive change according to the sample.

The rules were trained using the MATLAB trainlm function, and the Levenberg–MagqMardt rules were used to train the forward network. The absolute mean percentage error (MAPE) was used as the error criterion for testing the samples. As mentioned earlier, the BP model was built with 6 input neurons, 10 hidden layer neurons, and 1 output neuron; the learning step was 0.06, the number of training sessions was 1,000, and the acceptable error criterion was *ε*_0_=0.001.

The article "China's Economic Forecast Based on Machine Learning and Quantitative Easing" was published in 2022. Journal: Comput Intell Neurosci.

## 5. Case Studies

However, since the model has a 12-period lag in the decision variable, the valid sample is only 32 periods. The data relating to exports within the sample period are used as the training sample and the test sample (the first 26 periods are used as the training sample, which satisfies the sample size requirement of 3*∗k*+8, with *k* being the number of explanatory variables of 6. The last 6 periods are used as test samples).

After inputting the samples, the system learns by minimising the sum of squared errors between the desired output and the actual output, adjusting the weight matrix and the threshold vector. After 20 training sessions, the error of the model is reduced to within the required range and the system stops learning. By running the MATLAB program 1,000 times, the best network (i.e. the one with the lowest error) for the detection sample is obtained and used as the final model for the neural network method. The prediction results for the detection samples are shown in Figures 3 and 4.  Figure 5 shows that the model's predictions for China's exports to the USA are very close to the actual values, and the results are satisfactory. The average error of the normalized prediction sample is 0.0753, and the average error of the reduced prediction is 0.0365, which means that the theoretical deviation from the true value of exports predicted by the neural network method is no more than 3.65%.

Using this neural network, the forecast for September 2008 was US$22,967,000 thousand, which is 6.821% less than the true value of US$24,683,579 thousand. The forecast results are good.

## 6. Experimental Analysis

The ARIMA model is estimated based on the decision variables designed above. The first step is to check whether the original series of export values is stationary using the unit root test (ADF test). The results show that the export value series is smooth after first order differencing. Using the period January 2005 to August 2008 as the sample period, the model is estimated using EVIEWS software as follows:

(5) $$\begin{array}{c} \Delta {\text{EXPORT}}_{t}=143796.03-0.38^{*}\Delta {\text{EXPORT}}_{t-1}\left(0.679\right)\left(0.020\right),\\ \Delta ER_{t-1}\left(-1\right)+39.90^{*}\Delta {\text{GDP}}_{t-1}\left(-1\right)+29.34^{*}\Delta {\text{GDP}}_{t-1}\left(-12\right)-395211.46*,\\ \Delta {\text{IPI}}_{t-1}\left(-1\right)+\varepsilon_{t-1}\left(0.011\right)\left(0.108\right). \end{array}$$

Here, *ε*_*t*−1_ is the error term, which follows the standard normal distribution. The *p* values of the coefficients are in parentheses.

The article "China's Economic Forecast Based on Machine Learning and Quantitative Easing" was published in 2022. Journal: Comput Intell Neurosci.

The *p* values of the leading coefficients of ΔEXPORT_*t*−1_ and ΔGDP_*t*−1_ (0.050 and 0.108, respectively) are statistically significant at the 90% confidence level, suggesting that they should be used as determinants of the model. Other variables with larger *p* values are not statistically significant, but empirical experience shows that their impact on export value is not negligible.

Using the above model to forecast the value of China's exports to the USA over the sample period, the static forecast in EVIEWS is used.  Figure 6 shows a comparison between the predicted and true series of export values. It can be seen that the estimated ARMA model gives a better estimate of export values as the predicted values are derived from lagged decision variables. The mean absolute error of the model over the sample period is 5.503144%, which is greater than 3.65% predicted by the neural network approach for the test sample, which shows that the neural network approach outperforms the results predicted by the ARIMA model.

Based on this model, we can forecast one-period ahead, i.e., the export value for September 2008, using the sample data, and the forecast result is US$ 248,248,864,824, while the real export value is US$ 24,683,579,000, with an absolute error of 0.569%, which is very good. The ARIMA model outperforms the neural network approach in terms of this predictor.

Figure 7 shows a comparison of the AR(1)-GARCH model's predicted and real true value series for exports over the sample period, which is broadly similar to the ARIMA model. Here, the results are not analysed in detail.

The results of the three models are compared. The absolute mean percentage error (MAPE) is used as a comparison criterion to evaluate the fit and prediction of the three models:

(6) $$\begin{array}{c} \text{MAPE}=\frac{1}{n}\sum_{i=1}^{n}\left|\frac{\text{Export forecast value}-\text{export actual value}}{\text{Actual export value}}\right|. \end{array}$$

The prediction results of the three methods were compared with the true values for the six periods selected in the sample period and are tabulated as shown in Table 1.

A comparison of the forecast errors for each period for the three methods is tabulated in Table 2.

These two tables allow a comparison of the results of the three models, with the following conclusions. The BP neural network model best fits the export value in the test period with an average error of 3.65%, while the ARIMA and AR-GARCH models have similar results with an average error of 5.5% over the sample period, which is worse than the neural network method. However, the latter two models perform very well in terms of predicting export value over the forecast period, with a prediction error of 0.614% compared to 6.821% for the neural network method [15]. This is contrary to the thesis that the neural network method outperforms the time series method in both rice export and stock price forecasting. The author believes that this is due to the fact that different papers have studied different subjects, adopted different variables, and built different models. In the other papers, the nonlinearity of the neural network method, which does not take into account the seasonal term, is found to explain the fluctuation of export value better than the general linear method. As this paper takes into account the seasonal variables more than in the previous literature, it proposes to add lagged seasonal variables to the model to deal with seasonal effects so that the linear model is able to describe and fit the intrinsic regularity of export movements very well, while the neural network approach produces results that are more random and contingent than the linear model. In addition, as mentioned above, the ARIMA model based on the Bayesian search algorithm is less effective in predicting seasonal models than nonseasonal models, and it is suggested that the seasonal treatment in this paper can be used to compare the forecasting effectiveness of the models.

The article "China's Economic Forecast Based on Machine Learning and Quantitative Easing" was published in 2022. Journal: Comput Intell Neurosci.

## 7. Discussion

In the context of this paper, the author believes that there are three main ways for China to continue to steadily increase its exports to foreign countries in the context of the global economic crisis.

The government can provide subsidies to increase exports in two ways: firstly, by lowering the costs of enterprises to compensate for the higher export prices and stagnant sales caused by the appreciation of the RMB; secondly, by reducing the chances of losses and bankruptcy of Chinese enterprises through subsidies so that they, especially the powerful ones, can reserve their strength in the economic winter. However, as China has joined the WTO, many policies have to meet the requirements of the WTO, and the excessive use of the previous explicit subsidy policy will lead to many disputes. For example, research subsidies for high-tech enterprises: government investment in basic research projects in universities and government laboratories, followed by public procurement to support the initial application of these results in products and processes, which then spread to commercial applications [16, 17].

The economic crisis has led to a sharp decline in imports, but this is a structural reduction in demand, while demand for high-tech products is still high. The Chinese government should seize this feature and steadily promote the transformation and upgrading of China's export processing trade, encouraging enterprises to produce products with higher technological content, environmental protection and energy saving, and guiding the healthy development of advanced manufacturing and modern production-oriented services so as to identify and meet the new demands of foreign markets at a faster pace [18]. Steady industrial transfer between the east and the west: enterprises in the developed coastal areas of the south-east should transfer production links in the industrial chain to the central and western regions where the factors of production are less expensive and upgrade to higher value-added links such as design, R&D, and marketing. In this way, the comparative advantage of China's export sector in terms of price can be maintained in the face of the continued appreciation of the RMB [19].

The article "China's Economic Forecast Based on Machine Learning and Quantitative Easing" was published in 2022. Journal: Comput Intell Neurosci.

As export trade volumes are the result of a joint game between governments, especially China as a major exporter, they often lead to trade disputes. Therefore, while expanding its imports, China must also focus on a strategic approach and continue to strengthen and improve its international economic and trade relations [20]. For example, China can expand its foreign imports of products in demand at home, for example, by using China's large and risky dollar reserves to buy crude oil, minerals, and raw materials at lower prices and then sell them to the domestic market at lower prices, and by focusing on increasing imports of advanced technology, key equipment, and components [20].

## 8. Conclusions

The paper first uses six variables as determinants: export value, real exchange rate, Chinese GDP, US IPI, and their seasonal variables, and uses three methods: BP neural network, ARIMA, and AR-GARCH to model China's exports to the US and forecast the next period outside the sample interval. Then, the simulated results of the three models were compared with the real values for the sample period and the forecast period, using the absolute mean percentage error (MAPE) as the error indicator. The results show that all three models are able to simulate and predict China's exports to the US better. The BP neural network model is a good fit for the test period, while the ARIMA and AR-GARCH models have similar results, and they predict the forecast period very well. This is contrary to some papers which state that the neural network method is better than the time series method.

## Figures and Tables

**Figure 1:** Data on China's exports to the US over the sample period ($000s).

**Figure 2:** Summary of the variables determining the value of China's exports to the US.

**Figure 3:** Export prediction.

**Figure 4:** Comparison between the predicted and actual export values after reduction in the detection period of the neural network model export prediction versus actual value.

The article "China's Economic Forecast Based on Machine Learning and Quantitative Easing" was published in 2022. Journal: Comput Intell Neurosci.

**Figure 5:** Normalized predicted values for the detection period of the neural network model and after reduction predicted versus actual values.

**Figure 6:** ARIMA model sample period exports.

**Figure 7:** AR (1)-GARCH model sample period comparison of real and predicted export value series in the sample period.

**Table 1:** Comparison of predicted true values for each period obtained by the three methods.

	True value	Neural network method	ARIMA method	AR-GARCH method
2006.2	11218768	11948353	12060875	12135737
2007.2	16336347	17200569	15478242	16145578
2008.2	15475241	16253954	16754284	16886852
2008.5	21214314	21778439	21455741	27456721
2008.8	24035274	22788427	24451470	24574182
2008.9		22985700	24854741	24685231

**Table 2:** Comparison of the prediction errors obtained by the three methods for each period.

Method	Test sample period/sample period MAPE (%)	September 2008 forecast MAPE (%)
Neural network method	3.62	6.821
ARIMA method	5.503	0.57
GARCH method	5.582	0.614

## Data Availability

The experimental data used to support the findings of this study are available from the corresponding author upon request.
